The article "Antiproliferative Activity of Two Unusual Dimeric Flavonoids, Brachydin E and Brachydin F, Isolated from Fridericia platyphylla (Cham.) L.G.Lohmann: In Vitro and Molecular Docking Evaluation" was published in 2022. Journal: Biomed Res Int.

# Antiproliferative Activity of Two Unusual Dimeric Flavonoids, Brachydin E and Brachydin F, Isolated from *Fridericia platyphylla* (Cham.) L.G.Lohmann: *In Vitro* and Molecular Docking Evaluation

**DOI:** 10.1155/2022/3319203

**Published:** 2022-02-11

**Authors:** Carolina A. de Lima, Mayra C. Z. Cubero, Yollanda E. M. Franco, Carla D. P. Rodrigues, Jessyane R. do Nascimento, Débora B. Vendramini-Costa, Juliana M. Sciani, Cláudia Q. da Rocha, Giovanna B. Longato

**Affiliations:** ^1^Research Laboratory in Molecular Pharmacology of Bioactive Compounds, São Francisco University (USF), Bragança Paulista, SP, Brazil; ^2^Graduate Program in Health Science, São Francisco University, Bragança Paulista, SP, Brazil; ^3^Natural Products Chemistry Laboratory-Department of Chemistry-Federal University of Maranhão (UFMA), São Luís, MA, Brazil; ^4^Cancer Signaling and Epigenetics Program, Fox Chase Cancer Center, Philadelphia, PA, USA; ^5^Laboratory of Multidisciplinary Research, São Francisco University (USF), Bragança Paulista, SP, Brazil

## Abstract

Despite the breakthrough in the development of anticancer therapies, plant-derived chemotherapeutics continue to be the basis of treatment for most types of cancers. *Fridericia platyphylla* is a shrub found in Brazilian cerrado biome which has cytotoxic, anti-inflammatory, and analgesic properties. The aim of this study was to investigate the antiproliferative potential of the crude hydroethanolic extract, subfraction (containing 59.3% of unusual dimeric flavonoids Brachydin E and 40.7% Brachydin F), as well as Brachydin E and Brachydin F isolated from *F. platyphylla* roots. The cytotoxic activity was evaluated in glioblastoma, lung, prostate, and colorectal human tumor cell lines. The crude hydroethanolic extract did not present cytotoxic activity, but its subfraction presented lower IC50 values for glioblastoma (U-251) and prostate adenocarcinoma (PC-3) cell lines. Brachydins E and F significantly reduced cell viability, proliferation, and clonogenic potential of PC-3, inducing them to the process of regulated cell death. In silico studies have indicated nuclear receptors as targets for Brachydins E and F, and molecular docking has pointed out their binding into glucocorticoid receptor (GR) ligand pocket. Targeting GR pathway has been described as a therapeutic strategy, especially for prostate cancer. These results suggest that Brachydin E and Brachydin F are promising compounds to be further explored for their antitumor effects.

## 1. Introduction

Cancer is among the leading causes of death in the world, and according to the World Health Organization (WHO), 21.4 million new cases and 13.2 million deaths caused by cancer are expected by 2030 because of population growth and aging [1].

The article "Antiproliferative Activity of Two Unusual Dimeric Flavonoids, Brachydin E and Brachydin F, Isolated from Fridericia platyphylla (Cham.) L.G.Lohmann: In Vitro and Molecular Docking Evaluation" was published in 2022. Journal: Biomed Res Int.

There are many advances in diagnosis and treatment of different types of cancer, but there is still a need for new treatments, especially with decreased side effects. Chemotherapeutics of natural origin or derivatives of natural compounds have been widely used for the treatment of several types of cancer [2, 3]. According to the Brazilian Fund for Biodiversity (FUNBIO), Brazilian flora comprises about 55,000 described species, a number that represents 22% of world's total. Of note, plants from Cerrado, the second largest biome of Brazil, have been receiving increasing attention as sources of therapeutic agents, because secondary compounds from many of those plants are known to possess anticancer properties [4].

*Fridericia platyphylla* (Cham.) L.G.Lohmann (syn: *Arrabidaea brachypoda* Bureau, Bignoniaceae) is a shrub about 70 cm high found in Brazilian cerrado traditionally used for the treatment of renal calculi and inflammatory processes. According to the literature, *F. platyphylla* has medicinal properties, such as antifungal [5], anti-*T. cruzi* [6], antioxidant [7], anti-inflammatory [8], antimicrobial [7], analgesic [8], and leishmanicidal [9]. Studies recently published by our group showed that the phytochemical investigation of the hydroethanolic extract of its roots led to the isolation of several constituents: two glycosylated phenylethanoid derivatives, seven glycosylated dimeric flavonoids, being Brachydin E and Brachydin F, and other two compounds firstly described in the Bignoniaceae family, with no previous data in the literature about their pharmacological properties [9].

Considering the cytotoxic and antiproliferative activity recently described for the crude hydroethanolic extract of *F. platyphylla* in hepatocellular carcinoma and gastric adenocarcinoma cells [10], this study is aimed at investigating the in vitro antiproliferative effects of the crude hydroethanolic extract derived from *F. platyphylla* roots, hydromethanolic subfraction (containing 59.3% Brachydin E and 40.7% Brachydin F), and isolated compounds (Brachydin E and Brachydin F) in glioblastoma, lung, prostate, and colorectal human tumor cell lines. The isolated compounds from this species fit into a rare-structure group of dimeric flavonoids, because they are a result of the union of two chalcones, which highlight the importance of the present study.

## 2. Materials and Methods

### 2.1. Obtention of the Crude Hydroethanolic Extract, Subfraction, and Compounds Brachydins E and F

The crude hydroethanolic extract, subfraction, and compounds Brachydin E and Brachydin F were obtained as previously described by Rocha et al. [11]. After extraction, further liquid/liquid extractions with the hydroethanolic extract were carried out using CH_2_Cl_2_ (1 L) and H_2_O-MeOH (7 : 3) (1 L). The crude dichloromethanic (CH_2_Cl_2_) and hydromethanolic (H_2_O-MeOH) fractions were obtained after decantation and were evaporated to dryness under vacuum at approximately 40°C. The hydromethanolic fraction was initially fractionated by column chromatography (CC), using normal phase (silica gel), and a subfraction containing two compounds (59.3% Brachydin E and 40.7% Brachydin F) was obtained. The amount of each compound was given by the peak area on the HPLC-PDA. The subfraction was purified by CC. The fractions were combined according to the chemical composition determined by HPLC-PDA analysis, dried, analyzed by NMR, and properly stored, resulting in the isolation of high purity Brachydin E and Brachydin F. Chemical shifts are reported in parts per million (*δ*) using the residual CD_3_OD signal (*δ*_H_ 3.31) as the internal standard for both ^1^H NMR; the coupling constants (*J*) are reported in Hz.

The article "Antiproliferative Activity of Two Unusual Dimeric Flavonoids, Brachydin E and Brachydin F, Isolated from Fridericia platyphylla (Cham.) L.G.Lohmann: In Vitro and Molecular Docking Evaluation" was published in 2022. Journal: Biomed Res Int.

*Brachydin E*: ^1^H NMR (CD_3_OD, 500 MHz) *δ* 6.41 (1H, d, *J* = 2.2 Hz, H-2), 6.28 (1H, d, *J* = 2.2 Hz, H-4), 4.79 (1H, d, *J* = 11.3 Hz, H-6), 2.36 (1H, dd, *J* = 11.3, 2.6 Hz, H-6a), 3.26 (1H, d, *J* = 5.5 Hz, H-7), 6.38 (1H, d, *J* = 2.1 Hz, H-9), 6.30 (1H, d, *J* = 2.1 Hz, H-11), 5.34 (1H, d, *J* = 2.6 Hz, H-12a), 7.25 (2H, m, H-2′, 6′), 7.39 (3H, m, H-3′, 4′, 5′), 6.21 (1H, dd, *J* = 15.8, 5.5 Hz, H-*α*), 5.91 (1H, d, *J* = 15.8 Hz, H-*β*), 7.23 (2H, m, H-2^″^, 6^″^), 7.22 (2H, m, H-3^″^, 5^″^), 7.13 (1H, t, *J* = 7.0 Hz, H-4^″^), 3.85 (3H, s, 1-OMe), 3.67 (3H, s, 8-OMe), 3-GlcA: 4.94 (1H, d, *J* = 6.9 Hz, H-1′), 3.49 (1H, m, H-2′), 3.50 (1H, m, H-3′), 3.55 (1H, m, H-4′), 3.82 (1H, d, *J* = 7.6 Hz, H-5′), 10-GlcA: 4.97 (1H, d, *J* = 7.0 Hz, H-1′), 3.52 (2H, m, H-2′, 3′), 3.55 (1H, m, H-4′), 3.87 (1H, d, *J* = 7.6 Hz, H-5′) [11].

*Brachydin F*: ^1^H NMR (CD_3_OD, 500 MHz) *δ* 6.40 (1H, d, *J* = 2.1 Hz, H-2), 6.26 (1H, d, *J* = 2.1 Hz, H-4), 4.77 (1H, d, *J* = 11.3 Hz, H-6), 2.26 (1H, dd, *J* = 11.3, 2.4 Hz, H-6a), 3.23 (1H, d, *J* = 5.5 Hz, H-7), 6.36 (1H, d, *J* = 2.1 Hz, H-9), 6.29 (1H, d, *J* = 2.1 Hz, H-11), 5.32 (1H, d, *J* = 2.4 Hz, H-12a), 7.24 (2H, m, H-2′, 6′), 7.39 (3H, m, H-3′, 4′, 5′), 6.02 (1H, dd, *J* = 15.8, 5.5 Hz, H-*α*), 5.83 (1H, d, *J* = 15.8 Hz, H-*β*), 7.15 (2H, d, *J* = 8.8 Hz, H-2^″^, 6^″^), 6.77 (2H, d, *J* = 8.8 Hz, H-3^″^, 5^″^), 3.84 (3H, s, 1-OMe), 3.66 (3H, s, 8-OMe), 3.74 (3H, s, 4^″^-OMe), 3-GlcA: 4.94 (1H, d, *J* = 6.0 Hz, H-1′), 3.53 (2H, m, H-2′, 3′), 3.59 (1H, m, H-4′), 3.89 (1H, d, *J* = 9.5 Hz, H-5′), 10-GlcA: 4.98 (1H, d, *J* = 7.0 Hz, H-1′), 3.52 (2H, m, H-2′, 3′), 3.62 (1H, m, H-4′), 3.95 (1H, d, *J* = 9.6 Hz, H-5′) [11].

The article "Antiproliferative Activity of Two Unusual Dimeric Flavonoids, Brachydin E and Brachydin F, Isolated from Fridericia platyphylla (Cham.) L.G.Lohmann: In Vitro and Molecular Docking Evaluation" was published in 2022. Journal: Biomed Res Int.

### 2.2. Cell Culture

The biomonitoring of the crude ethanolic extract, subfraction, and compounds Brachydins E and F was performed by evaluating the cytotoxic activity in a panel of commercial human tumor cell lines purchased from the American Type Culture Collection—ATCC: 4 tumoral (U-251—glioblastoma, NCI-H460—lung, PC-3—prostate, and HT-29—colorectal) and 1 nontumoral (HaCat—keratinocyte).

### 2.3. Cytotoxicity Assay

For this assay, the colorimetric method 3-(4,5-dimethylthiazol-2-yl)2,5-diphenyltetrazolium bromide, MTT (Sigma) was used to indirectly evaluate cell viability by the mitochondrial enzymatic activity of living cells [12]. The cell suspensions were prepared in RPMI-1640 (Lonza) medium containing 5% FBS (Nutricell) and 1% PS (Nutricell). One hundred *μ*L of cell suspension containing 5000 cells was inoculated per well into 96-well plates and incubated for 24 hours at 37°C in a 5% CO_2_ atmosphere and humidity. After 24 hours, samples were diluted in DMSO and added to the cells at concentrations of 1.6, 3.12, 6.25, 12.5, 25, 50, and 100 *μ*g/mL (100 *μ*L/well) in triplicate and then incubated for 48 hours at 37°C in a 5% CO_2_ atmosphere and humidity. As a positive control, the chemotherapy drug doxorubicin hydrochloride, doxo (Eurofarma), was used at concentrations of 0.16, 0.31, 0.62, 1.25, 2.5, 5, and 10 *μ*g/mL (100 *μ*L/well) in triplicate. Final DMSO concentration (less than 1%) did not affect cell viability [13, 14]. After 48 hours of treatment, the treated cells were then stained with MTT. The absorbance data were analyzed and compiled in the graphs plotting the percentage of viable cells with the sample concentration. The IC50 (half maximal inhibitory concentration) values were calculated, which refers to the concentration of samples required to decrease in 50% cell viability. Isolated compounds Brachydins E and F, as well as doxorubicin, were also evaluated for the selectivity index (SI), which allows identifying the selectivity of the tested compounds for tumor lines in relation to the nontumoral cell line, therefore suggesting absence of potential side effects. In this study, SI was obtained from the following formula: IC50 of the nontumoral cell line (HaCaT)/IC50 of tumor cell lines. For this analysis, a SI value greater than or equal to 2.0 was adopted as significant, as previously described by the NCI, USA (National Cancer Institute, USA). By this assay, the PC-3 cell line (prostate) was chosen to continue the studies on antiproliferative activity.

### 2.4. Wound Healing Assay

This assay is widely used to study the characteristics of cell migration, as well as for the validation of molecules that might interfere with the proliferation process. For this assay, PC-3 cells were seeded in 6-well plates (COSTAR) at a density ranging from 5 × 10^5^ to 1 × 10^6^, and upon reaching 100% of confluence (about 24 hours), two slots were inserted in parallel within each well. Prior to treatments, four selected regions were photographed in a microscope with a coupled camera (Zeiss), and after that, treatments with DMSO, Brachydin E, and Brachydin F (at half IC50 concentration) were added. New images from the same regions were acquired over 24 and 48 hours after treatment. Moreover, the distance between the two margins of the slot was measured for each time point, using the ImageJ software 1.8.0_172(NIH). The results were expressed as percentage of slot closure, using the formula: (*A* initial distance–*A* final distance)/(*A* initial distance) × 100 = %of wound healing, being *A* is the measurement between the edges of the slot [15].

The article "Antiproliferative Activity of Two Unusual Dimeric Flavonoids, Brachydin E and Brachydin F, Isolated from Fridericia platyphylla (Cham.) L.G.Lohmann: In Vitro and Molecular Docking Evaluation" was published in 2022. Journal: Biomed Res Int.

### 2.5. Colony Formation Assay (Clonogenic Assay)

Colony formation or clonogenic assay is an *in vitro* quantitative technique to examine the capability of a single cell to grow into a large colony through clonal expansion. It was performed as described by Rajendran and Jain [16]. For this assay, 5000 cells were seeded in agar medium (Kasvi) in 6-well plates to prevent adherence of these cells to the well. Every three days, treatments with DMSO, Brachydin E, and Brachydin F (at half IC50 concentration) diluted in serum-free culture medium were performed. After 21 days in culture, the colonies were fixed by the gentle addition of 0.005% formaldehyde (Scientific Exodus) and stained with crystal violet (Nuclear). The wells were photographed, and the images were analyzed in the ImageJ software for quantification of the colonies.

### 2.6. Phosphatidylserine (PS) Externalization Assay

This test is based on the labeling with Annexin V-PE (phycoerythrin) and 7-amino-actinomycin D (7-Aminoactinomycin D-7-AAD), representing phosphatidylserine externalization (typically characteristic of regulated cell death, such as apoptosis) and loss of cell membrane integrity (typical of advanced cell death), respectively. Double negative cells are considered viable. PC-3 cells were inoculated into 6-well plates at density ranging from 1 × 10^5^ to 1 × 10^6^ cell/mL in RPMI medium +5% FBS and 1% PS and incubated at 37°C in a 5% CO_2_ atmosphere and humidity. After 24 hours of treatment with DMSO, Brachydin E, and Brachydin F (at half IC50 concentration), cells were trypsinized, and 100 *μ*L of the suspension was transferred to a round bottom 96-well plate and mixed with 100 *μ*L of Guava Nexin Reagent (Merck/Millipore) for 20 minutes in darkness. After that, the plate was analyzed on a GuavaEasyCyte 5HT Flow Cytometer Benchtop Flow Cytometer (Merck/Millipore).

The article "Antiproliferative Activity of Two Unusual Dimeric Flavonoids, Brachydin E and Brachydin F, Isolated from Fridericia platyphylla (Cham.) L.G.Lohmann: In Vitro and Molecular Docking Evaluation" was published in 2022. Journal: Biomed Res Int.

### 2.7. Molecular Docking

The target for molecular docking was selected in the RCSB PDB (Protein Data Bank)—accession codes 1A52 (chain A), 3OLS (all chains), 2V95, and 1A28 (chain A + B). OpenBabel Cheminformatics tool of ChemInfo (http://www.cheminfo.org/) was used to optimize the energy of the ligand (Brachydins), which was drawn and converted to PDBQT format, with 3D parameters and pH 7. The protein was prepared by removing missing atoms, chain breaks, and water molecules, and hydrogens were added considering pH 7.0. The grid was defined by 22 Å × 24 Å × 28 Å box centred in the central ligand position (cocrystal template for comparison). The analysis was conducted AutoDock Vina to get the binding energy (kcal/mol) and to the Chimera 1.15 software for distance calculation and amino acid bind determination.

### 2.8. In Silico Pharmacodynamics

Brachydins E and F structures were also submitted to SwissADME analysis, in order to verify the compounds' physico-chemical properties, solubility, lipophilicity, pharmacokinetics parameters (gastrointestinal and brain-blood barrier absorption and hepatic enzymes inhibition), and druglikeness, following the Lipinski's medicinal chemistry alert [17].

### 2.9. Statistical Analysis

Results were expressed as mean ± standard deviation (SD) of three independent experiments conducted in duplicate. Statistical analyses were performed with the GraphPad Prism 5 software. *t*-test and ANOVA followed by Tukey or Bonferroni post hoc test was used, and *p* values less than 0.05 were considered significant. For the cytotoxic activity assay, the linear regression of the curves was obtained using the mean growth percentage and calculated with the Origin software (OriginLab).

## 3. Results and Discussion

### 3.1. Phytochemical Analysis

The filtration and evaporation processes described in Section 2.1 resulted in 178.0 g of crude hydroethanolic extract. The hydromethanolic (H_2_O-MeOH) fractions were obtained after decantation and were evaporated to dryness under vacuum, yielding 66% of the dried fraction, respectively, based on the dry mass [11].

The high performance liquid chromatography-photo diode array-mass spectrometry (HPLC-PDA-MS) analysis of the hydromethanolic fraction revealed the presence of two compounds with ultraviolet-photo diode array (UV-PDA) spectra closely related to the dimeric flavonoids Brachydin E and Brachydin F [11]. According to the protonated molecular ions recorded in electrospray ionization mass spectrometry (ESI-MS), the mass weight was m/z 883 [M + Na]^+^ and m/z 913 [M + Na]^+^, respectively. The high-resolution- (HR-) ESIMS of Brachydin E and Brachydin F revealed a [M-H]- ion at m/z 859.2457 and 889.2586, respectively. All these data are in accordance with those described by Rocha et al. [11]. As shown in Figure 1, Brachydin E and Brachydin F are dimeric flavonoids differing among themselves only at the aromatic ring C by the presence of a methoxyl group in Brachydin F.

The article "Antiproliferative Activity of Two Unusual Dimeric Flavonoids, Brachydin E and Brachydin F, Isolated from Fridericia platyphylla (Cham.) L.G.Lohmann: In Vitro and Molecular Docking Evaluation" was published in 2022. Journal: Biomed Res Int.

The ^1^H NMR spectrum of Brachydin E revealed 13 aromatic protons, 2 ethylene units, 2 oxygenated methines, 2 aliphatic methines, and 2 methoxy groups. The different aromatic signals belonged to 4 independent rings named A, B, C, and D. A pair of meta-coupled protons at *δ*_H_ 6.41 and 6.28 (*J* = 2.2 Hz) was assigned to the protons H-2 and H-4 in the A ring. Similar to ring A, ring B exhibited another pair of meta-coupled protons at *δ*_H_ 6.38 and 6.30 (*J* = 2.1 Hz) attributed to H-9 and H-11. Two pairs of ortho-coupled protons at *δ*_H_ 7.25 (H-2′ and H-6′) and 7.39 (H-3′, H-4′, and H-5′) were assigned to ring C, while the remaining five aromatic protons corresponded to the unsubstituted ring D at *δ*_H_ 7.22 (H-3^″^ and H-5^″^) and 7.23 (H-2^″^ and H-6^″^). The presence of two *β*-glucuronic acids was revealed by their anomeric protons at *δ*_H_ 4.94 (1H, d, *J* = 6.0 Hz, 3-GlcA-H-1′) and 4.97 (1H, d, *J* = 7.0 Hz, 10-GlcA-H-1′). The NMR showed the presence of two free hydroxyl groups in Brachydin F [11].

### 3.2. Cytotoxic Activity of the Crude Hydroethanolic Extract, Fraction, and Isolated Compounds Brachydins E and F

The crude hydroethanolic extract did not present cytotoxic effect over none of the cell lines evaluated, but its subfraction reduced the IC50 values for glioblastoma (U-251) and prostate (PC-3) cell lines from 95.8 and 100 *μ*g/mL to 47.7 and 43.5 *μ*g/mL compared to the crude extract, respectively. The dimeric flavonoid Brachydins E and F isolated from this subfraction maintained the cytotoxicity for glioblastoma (U-251) and presented greater cytotoxic effects towards lung (NCI-H460) and prostate (PC-3) compared to the subfraction, and Brachydin E was more potent than Brachydin F for these cell lines as shown in Table 1 and Figure 2.

Moreover, the selectivity index (SI) values reveal that Brachydin E was 4 times more selective to prostate (PC-3) in comparison to HaCaT (nontumoral) than doxorubicin, a well-established chemotherapeutic agent (Table 2). Brachydin F SI value for PC-3 was almost equal to doxorubicin (Table 2). These results showed that Brachydins E and F isolated from Fridericia platyphylla present cytotoxic effects towards almost all cell lines tested, with selectivity to PC-3 cell lines, which prompted us to select this cell line for the subsequent studies with both compounds.

The article "Antiproliferative Activity of Two Unusual Dimeric Flavonoids, Brachydin E and Brachydin F, Isolated from Fridericia platyphylla (Cham.) L.G.Lohmann: In Vitro and Molecular Docking Evaluation" was published in 2022. Journal: Biomed Res Int.

### 3.3. Brachydins E and F Decreased Prostate PC-3 Cell Repopulation and Clonogenic Potential

As shown in Figure 3, a significant difference was observed between treatments: DMSO-treated cells (Figures 3(a), 3(b), 3(i), and 3(j)) managed to proliferate, repopulating 100% and 70.3% of the slot (Figures 3(e) and 3(m), respectively) after 48 h of treatment. Conversely, Brachydins E and F (Figures 3(c), 3(d), 3(k), and 3(l)) prevented cell repopulation, allowing only 20 and 13.2% of the slot to be closed after 48 h of treatment (Figures 3(e) and 3(m), respectively).

Data from the colony formation assay showed that Brachydins E and F were able to reduce the number of PC-3 cell colonies by over 68.9% and 60.1%, respectively, when compared to DMSO treatment over 21 days of experiment (Figures 3(f)–3(h) and 3(n)–3(p)). These results suggest that dimeric flavonoids Brachydins E and F prevent cell proliferation, which is in accordance with the cytotoxic activity observed above.

### 3.4. Brachydins E and F Induce Regulated Cell Death on PC-3 Cells

The phosphatidylserine externalization assay (Figure 4) showed that Brachydins E and F led to an increase of cells labeled with Annexin V (phosphatidylserine externalization) compared to treatment with DMSO, from 14.0 to 27.9 for Brachydin E (Figures 4(a)–4(c)) and from 13.6% to 25.9 for Brachydin F (Figures 4(d)–4(f)), with a consequent decline in viable cells (double negative labeling) from 79.1 to 68.7 for Brachydin E and from 75.1 to 62.5% for Brachydin F. There was no significant increase in the percentage of cells labeled only with 7-AAD, which means that cell membrane integrity was not compromised. These results suggest that the mechanism of action of this compound may involve induction of regulated cell death in PC-3 prostate cells, with cells in early cell death stage after 24 h of treatment.

### 3.5. In Silico ADME: Absorption, Distribution, Metabolism, and Excretion

Brachydins E and F were evaluated for their pharmacokinetics properties (Table 3). It was possible to observe that both molecules have similar physico-chemical characteristics. The only different parameters were LogP (partition coefficient), which was 3.02 for Brachydin E and 2.61 for Brachydin F and the TPSA (molecular polar surface area) values (251.36 A2 and 268.43 A2 for Brachydins E and F, respectively).

#### 3.5.1. Molecular Docking

Brachydins E and F were subjected to molecular docking analysis in order to find possible molecular targets for those ligands. Based on their structures, similar to steroids, and the results obtained by SwissTargetPrediction that indicated nuclear receptors as targets for Brachydins E and F (data not shown), estrogen (*α* and *β* subtypes), progesterone, and glucocorticoid receptors (Figure 5) were selected for the study.

The article "Antiproliferative Activity of Two Unusual Dimeric Flavonoids, Brachydin E and Brachydin F, Isolated from Fridericia platyphylla (Cham.) L.G.Lohmann: In Vitro and Molecular Docking Evaluation" was published in 2022. Journal: Biomed Res Int.

Table 4 shows the binding side, energy, interaction, and length for each Brachydin and their respective receptors. The glucocorticoid was the only receptor in which both molecules could bind in the ligand pocket. The same amino acids in which cortisol binds (Val17, Asp256, Lys359, Trp362) were found for Brachydins E and F, besides another residues that both Brachydins could bind. Brachydin E has a binding energy more favorable than Brachydin F (-9.56 and -8.68, respectively).

Moreover, considering the four binding amino acids, the bond length was shorter for Brachydin E, which means that ligand is positioned next to the protein target.

The ligand binding on other receptors (estrogen and progesterone), although with high blinding energy in some cases, did not occur in the pocket, with the binding taking place on the outside of the protein, in a region without biological significance. Figure 4 shows the target proteins and binding to ligand Brachydin E or F.

Natural products represent a rich source for the discovery and development of cancer preventive and anticancer drugs [18]. Despite the introduction of new drugs into the therapeutic arsenal of cancer, several tumors still lack adequate treatment. Natural sources are still available in abundance and offer the best possibilities of finding substances of therapeutic interest.

The Brazilian Cerrado is one of the major biogeographic regions of the world with more than 7000 native species of vascular plant. Many of these plants are commonly used as natural remedies by people living in this biome to treat several illnesses [13]. *Fridericia platyphylla* (Cham.) L.G.Lohmann (syn: *Arrabidaea brachypoda* Bureau, Bignoniaceae) is a native plant from Brazil, widely distributed in different biomes, but specially in cerrado, and the traditional use of teas prepared from the roots of this plant is already known for the treatment of kidney stone and arthritis [19]. Phytochemical studies have shown that plants of the genus *Arrabidaea* are sources of many compounds, including flavonoids [9].

The literature has shown that flavonoids are capable of inhibiting cell proliferation, tumor growth, and carcinogenesis. It has been widely reported that flavonoids interfere with the initiation, promotion, and progression of cancer by modulating different enzymes and receptors responsible for cell proliferation, differentiation, apoptosis, inflammation, angiogenesis, metastasis, and reversal of resistance to multiple drugs [20]. Currently, a new subclass of flavonoids, called biflavonoids (including dimeric flavonoids), has aroused scientific interest in this field. Because of their promising activities, these compounds could represent a great potential for drug development against many diseases, including cancer.

The article "Antiproliferative Activity of Two Unusual Dimeric Flavonoids, Brachydin E and Brachydin F, Isolated from Fridericia platyphylla (Cham.) L.G.Lohmann: In Vitro and Molecular Docking Evaluation" was published in 2022. Journal: Biomed Res Int.

Data on the antiproliferative activity of biflavonoids have been reported in the literature; however, it is still very limited. A study recently published has shown that the biflavonoid hinociflavone suppressed proliferation of colorectal tumor cells, induced apoptosis via the mitochondrial pathway mediated by the production of reactive oxygen species, and inhibited the migration/and invasion of tumor cells, proving that this biflavonoid can be used as an antitumor agent against colorectal cancer [21]. According to Yenesew et al. [22], the biflavonoid 7,7^″^-di-O-methylchamaejasmin isolated from the stem bark and roots of the Kenyan medicinal plant *Ormocarpum kirkii* S. Moore (Fabaceae) presented low values of IC50 for breast, colon, glioblastoma, human, and murine liver cancer cell lines, significantly elevating the number of cells in apoptosis in the sub-G0/G1 cell cycle phase and also causing cell cycle arrest in the G0/G1 phase. This compound altered the mitochondrial membrane potential (MMP) in acute lymphoblastic leukemia cells and caused an increase in reactive oxygen species generation. Therefore, these studies suggest that biflavonoids constitute an interesting class of compounds to be explored in cancer drug discovery and development.

The flavonoids Brachydin E and Brachydin F isolated from the crude hydroethanolic extract of *F. platyphylla* roots belong to the special group of natural compounds called dimeric flavonoids. The presence of chalcones in the Brachydin structures adds great pharmacological potential, since this group of substances has several pharmacological properties, such as antioxidant, cytotoxic, anticancer, antimicrobial, antiprotozoal, antiulcer, antihistamine, and anti-inflammatory activity. Some leading compounds with various pharmacological properties have been developed based on the chalcone skeleton [23].

In fact, our study describes the antiproliferative effect of two rare dimeric flavonoids, Brachydins E and F, isolated from the crude hydroethanolic extract of *F. platyphylla* roots and without any previous reports for their anticancer activities. Previous study published by our group has indicated that the flavonoids Brachydins A, B, and C, obtained from the root extract of *F. platyphylla* (Cham.) L.G. Lohmann, induce cytotoxicity in the human prostate tumor cell line PC-3 [10]. The difference between the compounds A, B, and C and Brachydins E and F is the presence of two *β*-glucuronic acids on the last two molecules.

The article "Antiproliferative Activity of Two Unusual Dimeric Flavonoids, Brachydin E and Brachydin F, Isolated from Fridericia platyphylla (Cham.) L.G.Lohmann: In Vitro and Molecular Docking Evaluation" was published in 2022. Journal: Biomed Res Int.

Herein, we show that Brachydin E and Brachydin F possess cytotoxic activity, with high selective index for the human prostate adenocarcinoma cell line PC-3. These results prompted us to select PC-3 for further studies. Taken altogether, the results obtained from the cytotoxicity assessment, wound healing, and clonogenic assay confirm the potent antiproliferative activity of Brachydins E and F for PC-3 cells, once these experiments revealed that these dimeric flavonoids are cytotoxic and inhibit cell proliferation. In agreement, the Annexin V-PE/7-AAD assay suggests that Brachydins E and F are leading prostate cells to death. Annexin V is a phospholipid binding protein with high affinity for phosphatidylserine that is located on the inner face of the plasma membrane of viable cells. In the early phase of some regulated cell death process, phosphatidylserine molecules are translocated to the outer face and free to bind to Annexin V, thereby labeling cells through PE. 7-AAD binds to cell DNA and acts as an indicator of membrane structural integrity since it is not able to label cells that are viable and in initial process of cell death [24]. Brachydins E and F decreased the percentage of viable cells and increased Annexin V labeling without interfering with the cell membrane structure of PC-3 cells, characteristic of an initial process of regulated cell death.

In an attempt to outline a possible molecular target for Brachydins, these molecules were subjected to molecular docking. This methodology is aimed at predicting the experimental binding modes and affinities of small molecules within the binding site of particular receptor targets and is currently used as a standard computational tool in drug design for lead compound optimization and in virtual screening studies to find novel biologically active molecules [25]. In silico studies have indicated nuclear receptors as targets for Brachydins E and F, and molecular docking has pointed out their binding into glucocorticoid receptor (GR) ligand pocket, at the same amino acids as cortisol [26]. It is known that glucocorticoid (GC) hormones exert an antiproliferative effect on various cells mediated by glucocorticoid receptor (GR), which acts as a transcription factor [27]. Targeting GR pathway has been described as a therapeutic strategy, especially for prostate cancer. Androgen (AR) and glucocorticoid (GR) receptor signaling plays opposing roles in prostate tumorigenesis: in prostate, AR acts as an oncogene, and GR is a tumor suppressor [28]. The glucocorticoid receptor (GR) is also hypothesized to participate in prostate therapy resistance [29]. This result suggests that Brachydins could interact with GR, which, in turn, leads to tumor suppression, culminating in apoptosis activation. In agreement with our study, Smith et al. [30] show that prostate tumor cell lines that lack AR (which is the case for PC-3) tend to express high levels of GR and that these cells were dependent on GR activity for their growth and survival. Further studies are necessary in order to confirm the relationship between Brachydins and GR and their downstream effects.

The article "Antiproliferative Activity of Two Unusual Dimeric Flavonoids, Brachydin E and Brachydin F, Isolated from Fridericia platyphylla (Cham.) L.G.Lohmann: In Vitro and Molecular Docking Evaluation" was published in 2022. Journal: Biomed Res Int.

Although Brachydins E and F differ among themselves only at the aromatic ring C (by the presence of a hydroxyl group in Brachydin E while Brachydin F presents a methoxyl group), results obtained in vitro have pointed out that Brachydin E has better potency in antiproliferative activity. To check their similarities and differences, an in silico absorption, distribution, metabolism, excretion (ADME) study was applied, which is an important tool for rational drug design [31]. Brachydins E and F have similar physico-chemical characteristics, with the exception of two parameters: Brachydin E has higher LogP and lower TPSA than Brachydin F. These findings indicate a better permeability through the plasma membrane for Brachydin E in comparison to Brachydin F, which can explain their different in vitro responses. Although the ADME study predicted low GI absorption for Brachydins E and F (suggesting in poor oral bioavailability), neither molecules have the potential to permeate the blood-brain barrier, which might indicate that they do not cause central nervous system (CNS) side effects.

Moreover, the ADME study also suggested that Brachydins E and F are not able to inhibit any metabolism enzyme, suggesting a lower risk for drug interaction [32].

The results herein described are very promising, considering that prostate cancer is the second most common neoplasm in the world among men, and the chemotherapy commonly used in the clinic for its treatment has extensive side effects such as neutropenia, thrombocytopenia, liver toxicity, fatigue, hypertension, and even leukemia induction [33–35]. Therefore, there is an intense search for new antineoplastic agents that are more powerful and have fewer side effects for the treatment of prostate cancer.

## 4. Conclusions

The collective reported data for dimeric flavonoids and the results obtained in our studies suggest that Brachydins E and F are promising compounds to be further explored for their antitumor effects. The results presented in this study for the dimeric flavonoids Brachydins E and F are unprecedented and reinforce the need for further studies on their mechanism of action, in view of the relevant antiproliferative property evidenced herein and the already reported antiproliferative properties of dimeric flavonoids.

The article "Antiproliferative Activity of Two Unusual Dimeric Flavonoids, Brachydin E and Brachydin F, Isolated from Fridericia platyphylla (Cham.) L.G.Lohmann: In Vitro and Molecular Docking Evaluation" was published in 2022. Journal: Biomed Res Int.

## Figures and Tables

**Figure 1:** Structures of the compounds isolated from *Fridericia platyphylla*.

**Figure 2:** Cell growth percentage after 48 h of treatment with Brachydin E (a), Brachydin F (b), doxorrubicin (c), extract (d), and subfraction (e). Human cell lines: U-251 (glioblastoma), NCI-H460 (lung, non-small-cells), PC-3 (prostate), HT-29 (colon), HaCat (keratinocytes, nontumoral).

**Figure 3:** Photomicrographs of PC-3 cells at 0 h (a, c, i, k) and after 48 h treatment with DMSO (b, j), Brachydin E (d), and Brachydin F (l). Percentage of wound closure for PC-3 cells over the treatment period (24 h and 48 h) with DMSO, Brachydin E, and Brachydin F, respectively (e, m). Photographs of PC-3 colonies treated with DMSO (f, n), Brachydin E (g), and Brachydin F (o) after 21 days. Number of PC-3 colonies formed after 21 days of treatment with DMSO, Brachydin E, and Brachydin F, respectively (h, p). ^∗∗^*p* < 0.01; ^∗∗∗^*p* < 0.001 ((e, m) ANOVA, Tukey test; (h, p) *t*-test).

**Figure 4:** Annexin V-PE/7-AAD data plots obtained for treatment with DMSO (a, d), Brachydin E (b), and Brachydin F (e). Number of cells (%) not labeled (double negative) or labeled with Annexin and 7-AAD, after 24 h of treatment with DMSO, Brachydin E (c), and F (f). ^∗^*p* < 0.05 (ANOVA, Bonferroni).

**Figure 5:** Molecular docking of Brachydins E and F and 4 different receptors: (a) ER-*α*/Brachydin E; (b) ER-*α*/Brachydin F; (c) ER-*β*1/Brachydin E; (d) ER-*β*1/Brachydin F; (e) glucocorticoid receptor/Brachydin E; (f) glucocorticoid receptor/Brachydin F; (g) progesterone receptor/Brachydin E; (h) progesterone receptor/Brachydin F.

**Table 1:** Mean and standard deviation of IC50 values for the crude hydroethanolic extract, subfraction, and isolated compounds obtained from *Fridericia platyphylla* roots in human tumor cell lines after 48 h of treatment.

IC_50_ (*μ*g.mL^−1^/*μ*M)	U-251	NCI-H460	PC-3	HT-29	HaCaT
Doxorubicin hydrochloride	>10/>17.2	>10/>17.2	1.0 ± 0.0/1.7 ± 0.0	>10/>17.2	2.1 ± 0.8/3.6 ± 1.3
Crude hydroethanolic extract	95.8 ± 0.0	>100	>100	>100	>100
Subfraction	47.7 ± 0.6	>100	42.5 ± 6.5	>100	>100
Brachydin E	55.7 ± 6.3/64.8 ± 7.3	23.4 ± 3.5/27.2 ± 4.0	5.9 ± 1.3/6.9 ± 1.5	96.9 ± 24.2/112.7	50.5 ± 6.8/58.7 ± 7.9
Brachydin F	44.1 ± 8.1/49.5 ± 9.1	88.7 ± 7.8/99.6 ± 8.7	33.1 ± 7.4/37.1 ± 9.2	>100/>112.4	59.9 ± 7.1/67.3 ± 7.9

IC_50_: half maximal inhibitory concentration; doxorubicin hydrochloride: positive control; human cell lines: U-251 (glioblastoma), NCI-H460 (lung, non-small-cells), PC-3 (prostate), HT-29 (colon), HaCat (keratinocytes, nontumoral).

The article "Antiproliferative Activity of Two Unusual Dimeric Flavonoids, Brachydin E and Brachydin F, Isolated from Fridericia platyphylla (Cham.) L.G.Lohmann: In Vitro and Molecular Docking Evaluation" was published in 2022. Journal: Biomed Res Int.

**Table 2:** Selective index values for doxorubicin hydrochloride (chemotherapy) and isolated compounds obtained from Fridericia platyphylla roots in human tumor cell lines after 48 h of treatment.

	U-251	NCI-H460	PC-3	HT-29
Doxorubicin hydrochloride	UD	UD	2.1	UD
Brachydin E	0.9	2.2	8.6	0.5
Brachydin F	1.4	0.7	1.8	UD

UD: undetermined. SI value greater than or equal to 2.0 was adopted as significant. Human cell lines: U-251 (glioblastoma), NCI-H460 (lung, non-small-cells), PC-3 (prostate), HT-29 (colon).

**Table 3:** Physico-chemical and ADME parameters predicted for Brachydins E and F.

Parameter	Brachydin E	Brachydin F
Hydrogen-bond acceptors (HBA)	16	17
Hydrogen-bond donors (HBD)	8	8
LogP	3.02	2.61
TPSA	251.36 A2	268.43 A2
Gastrointestinal absorption	Low	Low
Blood-brain barrier permeant	No	No
Metabolism enzyme inhibitors	0	0

**Table 4:** Binding site, energy, and site interaction of Brachydins to estrogen, glucocorticoid, and progesterone receptors.

Protein	PDB code	Binding site	Binding energy (kcal/mol)	Binding interaction	Bond length (A)
ER-*α*	1A52 (chain A)	Thr347 Asp351 Glu353			
Brachydin E			-6.65	LigO6-Lys362 LigO7-Leu372 LigO-Gln375	3.77 3.36 4.39
Brachydin F			-8.13	LigO16-Glu397 LigO3-Glu397 LigO4-Asn439 LigO6-Gln441	3.70 2.95 4.66 4.34
ER-*β*1	3OLS (all chains)	Glu305 Arg346 Phe356			
Brachydin E			-6.84	LigO4-Lys353 LigO11-Asp359 LigO5-Asp363 LigO7-Glu366	5.93 4.26 2.86 4.76
Brachydin F			-9.33	LigO13-Arg386 LigO14-Arg386 LigO9-Glu389	3.83 2.89 6.26
Glucocorticoid receptor	2 V95	Val17 Asp256 Lys359 Trp362			
Brachydin E			-9.56	LigO12-Val17 LigO5-Gln224 LigO5-Asp226 LigO9-Asp256 LigO4-Lys359 LigO11-Trp362	5.29 4.48 3.79 3.50 3.09 4.22
Brachydin F			-8.68	LigO3-Val17 LigO5-Asp256 LigC40-Lys260 LigO7-Lys359 LigO6-Trp362	3.74 3.04 4.33 5.71 3.59
Progesterone receptor	1A28 (chain A + B)	Gln725 Leu763 Arg766			
Bradychin E			-8.93	LigO6-Gln752 LigO15-Val730 LigO14-Gln747 LigO7-Glu911	3.78 3.89 3.46 2.82
Brachydin F			-8.08	LigO9-Glu723 LigO9-Ser898 LigO16-Glu904 LigO9-Ser910	9.37 4.81 3.82 3.54

## Data Availability

The data presented in this study are available on request from the corresponding author. The data are not publicly available due to privacy.
